# Antioxidant and Anticarcinogenic Potentials of Propolis for Dimethylhydrazine-Induced Colorectal Cancer in Wistar Rats

**DOI:** 10.1155/2022/8497562

**Published:** 2022-06-23

**Authors:** Alireza Salehi, Seyed Mohammad Hosseini, Sohrab Kazemi

**Affiliations:** ^1^Department of Pathology, Babol Branch, Islamic Azad University, Babol, Iran; ^2^Cellular and Molecular Biology Research Center, Health Research Institute, Babol University of Medical Sciences, Babol, Iran

## Abstract

Propolis is a natural compound with anticarcinogenic properties. The present study aimed to compare the inhibitory effect of ethanolic extract of propolis (EEP) and vitamin E on dimethylhydrazine-induced colon lesions in rats. In this study, 60 rats were randomly categorized into six 10-member groups. After 13 weeks, blood and colon tissue were sampled to examine some factors. The parameters included red (RBC) and white (WBC) blood cell profile, lactate dehydrogenase (LDH), C-reactive protein (CRP), total protein (TP), creatine kinase (CPK), and albumin, as well as the extent of colon histological lesions, protein expression (adenomatous polyposis coli (APC), proliferating cell nuclear antigen (PCNA), carcinoembryonic antigen (CEA), and platelet-derived growth factor (PDGF)), and oxidative stress markers (total antioxidant capacity (TAC), malondialdehyde (MDA), and superoxide dismutase (SOD)) in colon tissue. A significant decrease was observed in congestion, mitotic index, inflammation, and cell destruction in colon tissue in dimethylhydrazine group in comparison with the control group (*P* < 0.05). The EEP exposed rats exhibited a significant lower oxidative stress than the DMH group (*P* < 0.05). Furthermore, the extract significantly affected TAC level (*P* < 0.05). While the expression level of APC rose substantially in the EEP-treated group compared to the DMH group, the level of PCNA, CEA, and PDGF proteins significantly reduced. It seems that the EEP can efficiently prevent DMH-induced colonic lesions. Furthermore, its effectiveness is more than the vitamin E, which is a strong antioxidant.

## 1. Introduction

Cancer is considered one of the main factors of mortality and morbidity in the world [1]. Colorectal cancer (CRC) is the third most prevalent cancer among men and women in the USA [2], which in the development of the reactive oxygen species (ROS) level plays an important role. The high value of ROS affects several signaling pathways related to proliferation, tumor survival, invasion, and metastasis [3]. The body utilizes different mechanisms to modulate ROS concentration, one of which includes an antioxidant-based enzymatic system. In addition, peptic ulcers, necrosis, and inflammations are closely related to cancers in the organ [4]. Red blood cell (RBC) is the first body cell which reacts to irritating conditions such as stress. The oxidative stress of RBC is one of the reasons for disturbing its normal level [5], followed by other abnormalities and diseases like carcinogenicity [6, 7].

DMH causes lesions through two mechanisms, the first of which includes damage to mucus, and impairment in the uptake and output of substances, as well as the severe methylation of mucus. In the second mechanism, the balance between free radicals and the body's antioxidant power is disturbed [8]. The extent of tissue oxidative lesions can be generally estimated by measuring TAC and metabolites produced in the oxidation process (MDA) [9].

Propolis or bee glue is an organic sticky waxy substance produced by honey bees through mixing various secretions, plant pollen, beeswax, and saliva [10]. It, as a defense compound, protects the hive against different infections. In traditional medicine, this substance has been applied to treat various diseases and disorders worldwide [11]. Today, it is used in many studies because of having a wide range of medicinal properties like antimicrobial, antioxidant [12–14], and anti-inflammatory activities [15]. The antimicrobial potential of propolis can directly influence microorganisms, along with microbicidal properties through strengthening the immune system. Also, this compound can exhibit synergistic effects when consumed with antimicrobial drugs. Further, propolis enhances the activity of NK cells against cancer cells [11]. Recently, Masadah et al. [16] examined the effect of this substrate on breast cancer, and reported its antiproliferative, antimetastasis, and antioxidant activity, as well as its synergistic effect with radiotherapy and chemotherapy. A portion of the properties of ethanolic extract of propolis (EEP) is related to the existence of a substantial percentage of compounds such as chrysin and pinocembrin.

## 2. Method

### 2.1. Preparation of Propolis Extract

Propolis was collected from Mazandaran province in the north of Iran (52.35° E and 36.47° N). It was cut into smaller sections and dried at room temperature under shadow for two weeks [17], 500 g of which was added into 5 L of absolutely pure ethanol. After 72 hours, the extract was stored in sterilized microtubes at 4°C in a refrigerator until consumption [11].

### 2.2. Analysis of the Extract by Using Gas Chromatography-Mass Spectrometry (GC-MS)

The EEP was analyzed on a Shimadzu GCMS-TQ8040 NX to identify its different natural compounds. The spectrum of each component was compared to that of the compounds available in Wiley and NIST/EPA/NIH34-44 libraries and sorted based on its retention time in ascending order. The relative frequency of each substance was expressed based on its maximum. The structure of the detected natural compounds was drawn by using ChemDraw software. The values less than 1% were removed from the table [18].

### 2.3. Experimental Animals

A total of 60 eight-week-old male Wistar rats weighing 200-220 g were kept in the animal house of the Pasture Institute of Iran at 20-23°C and 60-70% relative humidity under a 12-h light/dark cycle. Additionally, the animals had access to a standard value of food and water during the experiment. The intended ethical protocols were respected at all stages of the study (IR.IAU.BABOL.REC.1399.102), and all animals were treated under the guidelines of the National Research Council and the ARRIVE guidelines 2.0 [19].

### 2.4. Study Design

Vitamin E and dimethylhydrazine (DMH) were purchased from Merck (Germany).

The rats were randomly divided into six 10-members groups. The first of which was the control group with no treatment and normal saline gavage. The second and third groups were, respectively, gavaged with 300 mg/kg of EEP [20] and 180 mg/kg of vitamin E [21] once a week. The weekly subcutaneous injection of DMH with a 30 mg/kg dose was applied for group four [22, 23]. Regarding the fifth and sixth groups, DMH-exposed animals received 300 mg/kg of propolis and 180 mg/kg of vitamin E, respectively.

At the end of 13 weeks, all rats survived, and were completely anesthetized intraperitoneally with a ketamine cocktail at 10 mg/kg concentration (10%, Bremer Pharma GmbH) and xylazine at 80 mg/kg level (2%, Alfasan Diergeneesmiddelen BV) [24], followed by weighting and sampling their blood. Then, colon tissue samples were taken, two portions of which were, respectively, placed in formalin for histological assessment and tissue homogenate preparation in a freezer at -80°C.

### 2.5. Blood and Serum Tests

The blood samples of the animals were poured in two separate tubes. A tube with EDTA was applied for taking a complete blood count(CBC) (Celltac Es MEK-7300K, Nihon Kohden). However, another tube containing no anticoagulant compound was centrifuged (Hettich®, model EBA 20) and used to determine serum markers on a BIOLIS24i autoanalyzer (Tokyo Boeki Medisys Inc.) [9].

### 2.6. Tissue Homogenization

In all groups, 0.25 g of colon tissue was homogenized in 1 mL of 50 mM phosphate buffer solution and 0.1 M EDTA with pH 7.4, and centrifuged at 4°C and 12000 rpm for 20 min. The supernatant was isolated and stored at -80°C until measuring oxidative stress markers. Protein content was determined in all homogenates by using Bradford assay [25] and bovine serum albumin as standard.

### 2.7. Malondialdehyde (MDA) Level Measurement

The Teb Pazhouhan Razi Kit was utilized for evaluating MDA level. For this purpose, the prepared tissue homogenate supernatant and reagents were brought to room temperature half an hour before starting the experiment. In the case of the presence of crystal, the reagents were heated to 50°C on a bain-marie and vortexed. The volume of thiobarbituric acid was doubled with deionized water, followed by mixing the reagents of HOAC (5×), alkali (10×), and thiobarbituric acid in a 1 : 1 : 2 ratio. Furthermore, 200 *μ*l of sample or standard was added into 800 *μ*l of working solution, and its lid was closed. The mixture was placed in a bain-marie at 95°C for 45 min, cooled in ice water containers rapidly, and centrifuged at 3000 rpm for 15 min. After transferring the samples to plate wells, their absorbance was read at 550 nm.

### 2.8. Determination of Superoxide Dismutase (SOD) Concentration

SOD concentration was examined by using SOD activity assay kit (Nasdox). Briefly, the tissue homogenate supernatant was prepared, and 50 *μ*l of sample and deionized water was poured into sample and control wells, respectively. Then, R1 and R2 were, respectively, added to both samples and controls. Following a room temperature incubation for 5 min in the absence of light, the absorbance of the mixtures was recorded at 405 nm.

### 2.9. Total Antioxidant Capacity (TAC) Assay

TAC was assessed with a TAC assay kit (Naxifer). After obtaining tissue homogenate supernatant, the reagents were placed at room temperature for 30 min; R2 solution was created by pouring 2.2 ml of R2b into each R2a bottle and vortexing completely until dissolution. Then, an equal value of the solution and R3 reagent was mixed and vortexed, to which R1 with five-fold volume was added. Finally, 5 *μ*l of sample or standard and 250 *μ*l of working solution were poured into each well, followed by evaluating optical absorbance at 593 nm after 5 min.

### 2.10. Protein Expression by Using Western Blot Analysis

During fixing a portion of colon tissues in 10% formalin buffer, 1 g of colon tissues from each group was frozen, lyzed with RIPA buffer, and subjected to a homogenizer (Tissue Mini Grinder, Model TD 1000) to achieve tissue homogenate. The homogenate was centrifuged at 12000 rpm for 10 min and western-blotted (Electrophoresis Western Blotting Tank, Model WPN-80). The blots were, respectively, incubated with the primary antibodies of APC, PCNA, CEA, and PDGF at 4°C for 12 h, and appropriate secondary ones related to peroxidase conjugate. In addition, *β*-actin antibody was applied as an internal control protein, relative to which the percentage of other antibodies was measured. The obtained membranes were washed with Tris-buffered saline(TBS) for 10 min and read by using PNP-1000D electrophoresis power supply. Ultimately, ImageJ software was utilized to analyze gray bar index [26, 27].

After determining the expression level of all proteins, the area under the diagram was calculated for each protein by using ImageJ software, and the ratio of the area to the *β*-actin protein was computed.

### 2.11. Histology

Regarding pathological examination, colon tissues were immediately rinsed with sterile normal saline and placed in 10% formalin buffer. Following tissue fixation (DS2080/H, Did Sabz Co.), osmotic dehydration and passage were performed, and paraffin blocks were prepared and cooled (TE100, Pouya Abzar Azma Model TE100). Then, the five-micron sections of tissues (DS4055, Did Sabz Co.) were H&E stained and examined on an Olympus CX23 optical microscope. In the histological analysis, Kruskal-Wallis and Mann–Whitney *U* assays were employed for the histopathological scoring between the groups, as well as determining mitotic index to compare the significance of their difference [28, 29].

### 2.12. Data Analysis

All of the data related to CBC, serum tests, and stress and inflammatory markers, as well as the ratios of western blot proteins, were analyzed by using SPSS 26 based on the one-way ANOVA and Duncan's post hoc tests. *P* < 0.05 was considered the main significant difference. The results are expressed as the mean ± standard deviation.

## 3. Results

### 3.1. Analysis of Propolis Ethanolic Extract through GC-MS

Based on the results, propolis ethanolic extract contained flavones, terpenes, flavonoids, and long chain fatty acids and exhibited high antioxidant and anti-inflammatory activity. The most important constituents of this extract included cinnamyl cinnamate [30], petroselinic acid [31], chrysin [32], pinocembrin [33, 34], and tetracosanoic acid [35], most of which have antioxidant, anti-inflammatory, and anticarcinogenic properties [33, 34] (Table 1).

### 3.2. Weight Changes

Table 2 presents the whole-body weights in all groups at the end of the 13th week. The DMH-exposed group lost a significant weight compared to the control group (*P* < 0.01). Meanwhile, it was observed that treating the DMH-exposed rats with the EEP elevated body weight significantly, as much as DMH + vitamin E-exposed rats, ended up at a better overall weight (Table 2).

### 3.3. Blood Parameters

The results revealed a decrease in RBC, WBC, RDW, MCHC, MCH, MCV, and hematocrit (HCT) level in the DMH group, but the differences between the groups were insignificant (Table 3).

### 3.4. WBC

Total WBC, neutrophil percentages, lymphocyte percentages, and platelet counts in all groups were measured. The total WBC counts significantly increased in the DMH group (*P* < 0.05) compared to the control group, while they significantly diminished in the EEP-exposed group (*P* < 0.05). The DMH group represented an increase in neutrophil percentage and a significant diminution in the lymphocyte percentage (*P* < 0.05), in both of which the EEP brought the number closer to that of the control (Table 4).

### 3.5. Biochemical and General Serum Inflammatory Marker

The results indicated that DMH increased serum total protein (TP) compared to control. However, serum albumin value, as the most characteristic protein, was not significantly different between the groups (Figure 1).

Other serum markers were enhanced in the DMH groups, among which CRP and LDH exhibited a significant rise (*P* < 0.0001). The consumption of EEP resulted in reducing the three markers, although no significant difference was found with the DMH group (Figure 1).

### 3.6. MDA Level in Colon Tissue

Regarding MDA level in colon tissue, a significant improvement was observed in the DMH group compared to the control group (*P* < 0.01), which declined among the rats treated with EEP, and a better response was achieved compared to the vitamin E (Figure 2).

### 3.7. SOD Concentration in Colon Tissue

As shown in Figure 1, SOD concentration is lower in the DMH group in comparison with the control group, while a significant increase was detected in the EEP-receiving group compared to the control group, DMH, and vitamin E-exposed groups. Also, there was a moderate rise in DMH + EEP group compared to the DMH group (*P* < 0.0001) (Figure 2).

### 3.8. TAC in Colon Tissue

The least and highest TAC were, respectively, related to the rats treated with DMH and EEP. Furthermore, both treatment groups revealed a significant promotion in this parameter in comparison with the DMH group (*P* < 0.0001 and *P* < 0.001, respectively) (Figure 2).

### 3.9. Protein Expression Level (Western Blot)

Based on the obtained ratios (Figure 3), the expression level of APC protein was significantly less in the rats exposed to DMH than the control group (*P* < 0.05), followed by a significant increase in the EEP-receiving group (*P* < 0.05). Regarding CEA protein, the expression level was significantly enhanced in the DMH group in comparison with the control (*P* < 0.05), which significantly diminished in the EEP-treated group (*P* < 0.05). Compared to the control group, a significant rise was detected in the DMH group in terms of PCNA protein expression (*P* < 0.05). However, both treatment groups experienced a significant reduction in this regard compared to the DMH group (*P* < 0.05), in which EEP led to significantly better outcomes than the vitamin E (*P* < 0.05). Finally, the results indicated the significantly greater expression level of PDGF protein in the DMH group compared to the control group, which significantly declined in both treatment groups (*P* < 0.05) although their difference with the control group was insignificant (Table 5).

### 3.10. Histological Observations

Characteristic pathological lesions such as mitotic index, inflammatory cell infiltration level, and necrosis were scored and compared between various groups (as the average number of mitoses in 10 HPF at the tumor area [28]) (Figure 4).

The ACF, the necrosis, inflammatory cells, and mitotic levels were not significantly different in the control, EEP, and vitamin E-exposed groups. However, a significant difference was observed between DMH group with the controls in terms of all four markers (*P* < 0.05). The EEP-treated group experienced a significant diminution in the number of ACF, necrosis, and mitotic index compared to the DMH group (*P* < 0.05) (Table 6).

## 4. Discussion

The simultaneous administration of EEP by gavage and DMH by injection led to reduced inflammatory and anticarcinogenic properties during the precarcinogenesis and pretumorigenesis phases in colorectal tissue. Overall, the EEP decreases tissue oxidative stress and reduces the inflammation in precarcinogenesis phase. Additionally, it positively regulated the expression of CEA, PCNA, APC, and PDGF proteins and substantially affected blood and serum factors. No adverse effect was found in the Wistar rats following the consumption of EEP. As already mentioned, the rats receiving 30 mg/kg of DMH [36] were treated with EEP and vitamin E for 13 consecutive weeks. It seems that chrysin and pinocembrin were responsible for the therapeutic power of the extract in this study. Chrysin is considered as a natural flavone with antioxidant, anti-inflammatory, and anticarcinogenic potentials [32], which seemed had led to decreased mitotic index in colon tissue. Further, pinocembrin represents antioxidant, anticarcinogenic, antitumor, and antimicrobial activities, leading to cancer cell apoptosis and tumorigenesis prevention. These two compounds can be utilized in anticancer combination drugs [33].

The rat's weight can change during a lot of diseases [37, 38]. Based on the results of the previous studies [39–43], DMH and its metabolites as a carcinogen induce the different levels of inflammation, precancerous, weight loss [44], and cancerous lesions. Weight loss is associated with the colon cancer [45], and the main possible reason for the weight loss would be the reduced function of the colon epithelium, which mainly caused by a wide inflammation that led to a lower absorption of feed [44]. Dolara et al. [46] proved the ability of oral antioxidants to diminish the effects and lesions induced by DMH. In the present study, the use of DMH negatively affected RBC, WBC, and stress levels, which is consistent with the results of Jrah et al. [47] concerning the effect of *Nigella sativa* on the DMH-caused lesions.

Since DMH leads to free radical generation in blood and oxidative stress in erythrocytes, a therapeutic compound should have high antioxidant activity to reduce free blood antioxidants for preventing oxidative stress in erythrocytes [48–51]. This surge in stress disturbs the immune system [52]. That could be the result of inflammation or furthermore, the reflection of tumorigenesis and neoplasm, to cope with which phagocyte and lymphocyte percentage promote with more rate due to the body's need [53, 54]. Regarding the present study, WBC level elevated in the DMH group, while a decrease in RBC was examined (Tables 2 and 3), which are both supported by the results of previous studies which revealed that lipid peroxidation leads to interference in erythrocyte function (e.g., [55]).

The consumption of DMH significantly enhanced CRP and LDH compared to the control (*P* < 0.05). In terms of CPK level, a rise was obtained in the DMH group compared to the control, which may be ascribed to skeletal muscle and liver problems, heart damage, and myocardial infarction. An elevated CRP level as an inflammatory biomarker following the use of DMH represents the body's acute phase [56]. In this regard, the results of the present study indicated a significantly less CRP level in the EEP-treated group, resulted by demonstrating an improvement in general conditions and a decline in tissue inflammation. Furthermore, the significant promotion in LDH level, as an enzyme existing in most of the live cells, exhibits extensive destructions at cellular level [57, 58]. This parameter significantly diminished after using the EEP, which may be due to less cell destruction (Figure 1).

The utilization of DMH resulted in significant changes in the concentrations of three tissue stress markers significantly (*P* < 0.05). The changes in oxidative stress markers are consistent with the pathological observations of the colon. Further, a decrease was found in the SOD level, as an antioxidant enzyme, in the DMH group compared to the control group [59]. Lipid peroxidation products such as MDA are known as oxidative stress biomarkers for determining the extent of cell damage [60, 61], which significantly increased in the DMH group compared to the control group (*P* < 0.05), by causing cell damages. Similarly, Lokeshkumar et al. [62] reported high lipid peroxidation in colon tissue following the use of DMH. That issue is in line with the result of the present study which suggested that lipid peroxidation products had irritative effects and enhanced secondary neoplasm rate, along with causing oxidative stress [63]. The previous studies have revealed that reduced TAC diminishes the body's ability to cope with oxidative stress and accelerates the peroxidation-caused lesions [64, 65]. Due to the great antioxidant properties of EEP, it elevated TAC level significantly in EEP-treated group compared to the DMH group (*P* < 0.05), and improved the power of the body's antioxidant system against free radicals and metabolites created in lipid peroxidation cycle. The pathological assessments and some serum markers, as the general indices of inflammation and cell damages, can help to diagnose and determine more accurate prognosis (Figure 3) [66]. Overall, these results are consistent with the previous studies, which have shown propolis as an antistress agent [67, 68].

Moreover, the use of DMH caused various tissue lesions in Wistar rat colon, which is in line with the results of the previous studies [69, 70]. The most typical incidence in DMH-induced rats is the ACFs [71, 72], which was reduced by treating the rats with the EEP. The number of ACF in DMH group showed the precancerous phase in the colon tissue, while in the EEP-treated group, the ACF number was reduced significantly(*P* < 0.0001). The DMH-exposed cells exhibited necrosis signs, a rise in mitotic index, and inflammatory cell infiltration due to methylation and promoted free radicals in the tissue [73], after scoring and classifying occurred lesions [29, 74, 75]. Compared to the DMH group, mitotic index and necrosis were significantly reduced in the EEP-exposed group because of decreasing free radicals due to a decline in lipid peroxidation in colon tissue (*P* < 0.05) (Table 6).

Regarding the expression level of CEA protein, a significant rise was detected in the DMH group compared to the control group (*P* < 0.05), which indicated the cancerous status of tissue, since the enhanced CEA content is a colorectal cancer-specific marker [76]. The CEA is a glycoprotein created during embryonic stage, and its production stops after birth [77]. The CEA concentration in serum is low, which significantly improves in adults when developing cancer. Additionally, tumor cell secretions elevate CEA level [78]. In this study, the DMH led to a disruption in the oxidant balance of colon tissue, followed by methylation, mutation, and carcinogenesis in tissue. The microtumors of the tissue increase CEA content, which significantly diminished in the EEP-receiving group compared to the DMH group because of eliminating the primary cause of the carcinogenetic cascade of DMH (oxidant balance of the tissue). Another protein under study, PCNA, is an antigen for cell nucleus proliferation, which acts as a DNA clamp as a factor for DNA polymerase in eukaryotic cells, and is essential for proliferation. The synthesis and expression of PCNA promote in proliferating cells [79], which represents cell proliferation and is considered as a reliable index for evaluating tumor cell proliferation [80]. The results of the present study revealed higher PCNA expression in all DMH-exposed groups compared to the control. Interestingly, the EEP prevented cells, especially cancer cells, from over-proliferating in comparison with the DMH group. In other words, the EEP exerts its antitumor potentials through inhibiting cancer cell proliferation. The reduction in APC protein concentration, caused by chromosomal instability, helps to form tumor since the protein acts as a brake for cell divisions [81]. In terms of APC level, a significant decrease was observed in the DMH group compared to the control group (*P* < 0.05), by representing the loss of chromosomal stability, followed by a promotion in unbridled cell divisions and cell tumorigenesis. Furthermore, the EEP elevated the reexpression of APC gene, enhanced APC protein concentration in cells, and consequently improved chromosomal stability to control cell reproduction cycle and diminish tumorigenesis rate. The PDGF is one of the cell division and growth factors, the expression of which increases the uncontrollable cell growth and tumorigenesis in cancers and tumors [82, 83]. This factor causes cancer cell metastasis [84]. Based on the results of the present study, PDGF significantly rose in the DMH group compared to the control group (*P* < 0.05), which significantly declined in the EEP-treated group. PDGF is a cancer marker, which is likely decreased due to the inhibition of its production. The clinical manifestation of its reduction included a decrease in the congestion observed in histology and a reduction in PDGF protein level in colon tissue (Table 4). This result is consistent with that obtained by Okda et al. [85] which demonstrated greater PDGF and CEA content after consuming the DMH and declined PDGF following the use of indometacin-vitamin D combination as therapeutic factors.

## 5. Conclusion

The ethanolic extract of propolis at 300 mg/kg can efficiently reduce oxidative stress through controlling lipid peroxidation pathway due to its anti-inflammatory, anticarcinogenic, antitumor, and antioxidant properties. This extract significantly elevates the power of the body's antioxidant defense system, leading to a diminution in free radicals. It also results in lower uncontrollable cell division rate, as well as a decreased rate and extent of carcinogenesis and tumorigenesis through controlling cell division markers.

## Figures and Tables

**Figure 1:** Comparison between general serum biochemical indices. ∗*P* < 0.05, ∗∗*P* < 0.01, ∗∗∗*P* < 0.001, and ∗∗∗∗*P* < 0.0001: significant compared to the DMH group. All results are expressed as the mean ± standard deviation. *n* = 10.

**Figure 2:** MDA, SOD, and TAC levels in the different groups. ∗∗*P* < 0.01, ∗∗∗*P* < 0.001, and ∗∗∗∗*P* < 0.0001: significant compared to the DMH group. All results are expressed as the mean ± standard deviation. *n* = 5.

**Figure 3:** Protein expression after western blot analysis of the colon tissues in gray scale.

**Figure 4:** Comparison of colon tissue indices of the different groups. Normal tissue presents in the control, EEP, and vitamin E groups. ACF (aberrant crypt foci) with dysplasia is shown with the left arrow. The epithelium displays nuclear stratification with rounded nuclei and hyperchromatic nucleoli. There is marked depletion of goblet cells in the dysplastic crypts. Necrosis (right arrow), mitosis (up arrow), and inflammatory cells infiltration (stars) are observed in DMH and therapeutic groups. Magnification 10× and 40×, H&E stain.

**Table 1:** Results of analyzing EEP by using GC-MS.

Chemical constituents	RT	Peak area (%)	MW (mg/Mol)	MF
Rosifoliol	15.315	1.35	222.37	C_15_H_26_O
Petroselinic acid	20.097	1.30	282.46	C_18_H_34_O_2_
Cis-ferulic acid	21.281	1.07	194.18	C_10_H_10_O_4_
7-Methylchrysin	22.482	11.63	268.26	C_16_H_12_O_4_
Cinnamyl cinnamate	22.627	3.39	264.3	C_18_H_16_O_2_
Pinocembrin	23.348	15.28	256.25	C_15_H_12_O_4_
Benzyl ferulate	23.897	1.66	284.31	C_17_H_16_O_4_
Hexadecane	24.503	1.10	226.44	C_16_H_34_
Chrysin	25.017	2.40	254.24	C_15_H_10_O_4_
Tetracosanoic acid	25.087	18.09	368.63	C_24_H_48_O_2_
1-Docosene	25.849	2.01	308.6	C_22_H_44_
Octacosyl acetate	27.778	3.84	452.8	C_30_H_60_O_2_
(Z)-9-tricosene	27.865	1.95	322.6	C_23_H_46_
1-Pentacosene	30.729	9.48	350.7	C_25_H_50_

**Table 2:** Comparison between the whole-body weights of each group at the end of the 13th week. Weight changes between the groups are compared with the control group. Significant differences between the groups are shown with different letters from the highest to the lowest (a, b, c, d, e). All results are expressed as the mean ± standard deviation. *P* < 0.01. *n* = 10.

Groups	Initial week (g)	Final week (g)	Weight change (%)
Control	203 ± 1.58	357.60 ± 7.83^b^	
EEP	204 ± 3.16	386.60 ± 12.22^a^	+8.11
Vitamin E	205 ± 2.55	360.40 ± 7.06^b^	+0.78
DMH	202 ± 0.71	252.80 ± 5.07^e^	-29.31
DMH + EEP	203.80 ± 2.59	297 ± 10.3^c^	-16.95
DMH + vitamin E	202.40 ± 1.34	277.20 ± 10.31^d^	-22.48

**Table 3:** Comparison between CBC parameters in each group. All results are expressed as the mean ± standard deviation. *n* = 10.

Groups	RBC (×10^6^/*μ*l)	HGB (g/dl)	HCT (%)	MCV (fL)	MCH (pg)	MCHC (g/dl)	RDW (%)
Control	8.12 ± 0.63	13.64 ± 1.26	40.7 ± 4.14	51.06 ± 2.22	17.16 ± 0.97	33.56 ± 0.68	14.35 ± 1.00
EEP	8.2 ± 1.11	13.6 ± 1.03	39.75 ± 3.23	52.01 ± 2.38	17.21 ± 0.79	33 ± 1.62	14.2 ± 0.73
Vitamin E	8.32 ± 0.55	14.15 ± 0.76	41.2 ± 5.77	50.24 ± 1.41	17.08 ± 0.98	33.6 ± 1.34	13.76 ± 0.9
DMH	7.54 ± 1.06	12.94 ± 1.33	39.19 ± 5.03	49.43 ± 4.76	16.99 ± 0.81	32.44 ± 0.94	13.76 ± 0.69
DMH + EEP	7.97 ± 0.84	13.05 ± 1.00	38.58 ± 3.07	50.23 ± 2.04	16.94 ± 0.45	32.69 ± 1.33	14.34 ± 0.66
DMH + vitamin E	8.09 ± 0.67	13.24 ± 1.12	39.88 ± 4.37	49.51 ± 2.45	17.11 ± 0.69	33.59 ± 1.82	13.61 ± 1.1

**Table 4:** Comparison between WBC and platelet. ∗*P* < 0.05: significant compared to the DMH group. All results are expressed as the mean ± standard deviation. *n* = 10.

Groups	WBC (×10^3^/*μ*l)	Neutrophil (%)	Lymphocyte (%)	Platelets (×10^3^/*μ*l)
Control	7.93 ± 1.24∗	57.83 ± 10.29∗	45 ± 10.16∗	734 ± 67.44
EEP	7.89 ± 1.03	59.86 ± 11.87	43.31 ± 11.45∗	769.25 ± 117.87
Vitamin E	7.6 ± 1.36	64.16 ± 11.62	42.21 ± 7.68∗	791.13 ± 65.42
DMH	9.58 ± 2.12	72.4 ± 14.28	26.93 ± 8.38	786.63 ± 146.48
DMH + EEP	7.93 ± 1.99	68.28 ± 10.65	31.3 ± 6.26	778 ± 100.67
DMH + vitamin E	8.2 ± 1.36	70.53 ± 8.99	29.71 ± 7.81	803.63 ± 93

**Table 5:** Comparison between the expression level of proteins relative to that of *β*-actin in colon tissue. ∗*P* < 0.05: significant compared to the DMH group. All results are expressed as the mean ± standard deviation. *n* = 4.

Groups	APC	CEA	PCNA	PDGF
Control	0.99 ± 0.05∗	0.39 ± 0.03∗	0.72 ± 0.08∗	0.98 ± 0.26∗
DMH	0.62 ± 0.05	0.82 ± 0.21	1.49 ± 0.15	1.38 ± 0.12
DMH + EEP	0.80 ± 0.12∗	0.61 ± 0.10∗	0.86 ± 0.05∗	0.85 ± 0.11∗
DMH + vitamin E	0.65 ± 0.14	0.71 ± 0.09	1.02 ± 0.12∗	0.94 ± 0.08∗

**Table 6:** Comparison between the tissue inflammation, mitotic, and necrosis indices of the different groups. *P* values less than 0.0001 were considered statistically significant. All results are expressed as the mean ± standard deviation. *n* = 6.

Group	ACF (number/cm^2^)	Mitosis	Inflammatory cells infiltration	Necrosis
Control	0	0.3 ± 0.32	0.1 ± 0.1	0.2 ± 0.14
EEP	0	0.1 ± 0.16	0.1 ± 0.1	0.1 ± 0.11
Vitamin E	0	0.2 ± 0.22	0.1 ± 0.1	0.1 ± 0.12
DMH	28.4 ± 2.61^a,e,f^	20.7 ± 1.18^a,e,f^	1.9 ± 0.35^a^	2.1 ± 0.27^a,e,f^
DMH + EEP	14.6 ± 1.6^b,e,g^	10.1 ± 1.11^b,e,g^	1.2 ± 0.41	1.1 ± 0.25^b,e^
DMH + vitamin E	20.4 ± 1.57^c,f,g^	16.7 ± 1.34^c,f,g^	1.3 ± 0.38	1.2 ± 0.26^c,f^

^a^Statistically significant differences between control and DMH treated observed. ^b^Statistically significant differences between control and DMH + EEP-treated observed. ^c^Statistically significant differences between control and DMH + Vit E-treated observed. ^e^Statistically significant differences between DMH and DMH + EEP-treated observed. ^f^Statistically significant differences between DMH and DMH + Vit E-treated observed. ^g^Statistically significant differences between DMH + EEP and DMH + Vit E-treated observed.

## Data Availability

Data are available on the request from the corresponding author.

## Abbreviations

DMH: Dimethylhydrazine
EEP: Ethanolic extract of propolis
CRC: Colorectal cancer
RBC: Red blood cell
WBC: White blood cell
LDH: Lactate dehydrogenase
CRP: C-reactive protein
TP: Total protein
CPK: Creatine kinase
APC: Adenomatous polyposis coli
PCNA: Proliferating cell nuclear antigen
CEA: Carcinoembryonic antigen
PDGF: Platelet-derived growth factor
TAC: Total antioxidant capacity
MDA: Malondialdehyde
SOD: Superoxide dismutase
ROS: Reactive oxygen species
NK Cells: Natural killer cells
HPLC: High-performance liquid chromatography
GC-MS: Gas chromatography mass spectrometry
EDTA: Ethylenediaminetetraacetic acid
CBC: Complete blood count
RDW: Red cell distribution width
MCHC: Mean corpuscular hemoglobin concentration
MCH: Mean corpuscular hemoglobin
MCV: Mean corpuscular volume.
